# Performance on the Frontal Assessment Battery is sensitive to frontal lobe damage in stroke patients

**DOI:** 10.1186/1471-2377-13-179

**Published:** 2013-11-16

**Authors:** Bruno Kopp, Nina Rösser, Sandra Tabeling, Hans Jörg Stürenburg, Bianca de Haan, Hans-Otto Karnath, Karl Wessel

**Affiliations:** 1 Cognitive Neurology, Technische Universität Braunschweig, Salzdahlumer Str. 90, Braunschweig 38126, Germany; 2 Department of Neurology, Braunschweig Hospital, Salzdahlumer Str. 90, Braunschweig 38126, Germany; 3 Department of Neurology, Hannover Medical School, Carl-Neuberg-Str. 1, Hannover 30625, Germany; 4 Klinik Niedersachsen, Hauptstr. 59, Bad Nenndorf 31542, Germany; 5 Division of Neuropsychology, Center of Neurology, Hertie-Institute for Clinical Brain Research, University of Tübingen, Hoppe-Seyler-Str. 3, Tübingen 72076, Germany; 6 Department of Psychology, University of South Carolina, 915 Greene Street, Columbia SC 29208, USA

**Keywords:** Frontal assessment battery (FAB), Abstraction, Fluency, Response inhibition, Anterior insula

## Abstract

**Background:**

The *Frontal Assessment Battery* (*FAB*) is a brief battery of six neuropsychological tasks designed to assess frontal lobe function at bedside [Neurology 55:1621-1626, 2000]. The six *FAB* tasks explore cognitive and behavioral domains that are thought to be under the control of the frontal lobes, most notably conceptualization and abstract reasoning, lexical verbal fluency and mental flexibility, motor programming and executive control of action, self-regulation and resistance to interference, inhibitory control, and environmental autonomy.

**Methods:**

We examined the sensitivity of performance on the *FAB* to frontal lobe damage in right-hemisphere-damaged first-ever stroke patients based on voxel-based lesion-behavior mapping.

**Results:**

Voxel-based lesion-behavior mapping of *FAB* performance revealed that the integrity of the right anterior insula (BA13) is crucial for the *FAB* global composite score, for the *FAB* conceptualization score, as well as for the *FAB* inhibitory control score. Furthermore, the *FAB* conceptualization and mental flexibility scores were sensitive to damage of the right middle frontal gyrus (MFG; BA9). Finally, the *FAB* inhibitory control score was sensitive to damage of the right inferior frontal gyrus (IFG; BA44/45).

**Conclusions:**

These findings indicate that several *FAB* scores (including composite and item scores) provide valid measures of right hemispheric lateral frontal lobe dysfunction, specifically of focal lesions near the anterior insula, in the MFG and in the IFG.

## Background

The *Frontal Assessment Battery* (*FAB*) is a brief battery of six neuropsychological tasks that was specifically designed to assess frontal lobe function at bedside [1]. The historical roots of the six *FAB* tasks can be found in the careful observation of dysexecutive behavior in patients with frontal lobe lesions, pioneered by Luria [2], Lhermitte, Pillon, and Serdaru [3], and others in the second half of the 20th century. The six *FAB* tasks explore cognitive and behavioral domains of executive functioning that are thought to be critically dependent on the integrity of the frontal lobes. The use of the *FAB* is becoming increasingly popular for a variety of applications in neurology, most notably the early diagnosis of neurodegenerative dementing diseases such as the behavioral variant of fronto-temporal lobar degeneration (bvFTLD; [4,5]). The *FAB* is easy to administer, requires less than ten minutes to complete, and is well accepted by patients. The reported psychometrics of *FAB* reliability and validity are satisfactory [1], yet the anatomical correlation between *FAB* scores and frontal lobe damage has never been established in studies of stroke patients. The claim that the *FAB* yields indices of frontal lobe damage was derived from data obtained with similar tasks, but never from the *FAB* tasks themselves [1].

In the present study, we investigated the sensitivity of performance on the *FAB* to frontal lobe damage in stroke patients using voxel-based lesion-behavior mapping (VLBM; [6-8]). In contrast to traditional overlap designs of neuropsychological patient groups [9], voxel-based lesion-behaviour analysis yields a sophisticated statistical approach to uncover brain-behaviour relationships. Voxelwise statistical analysis objectively estimates which brain regions indeed are associated with behavioral deficits without any prior categorization of stroke patients into, e.g., groups with more anterior versus more posterior brain damage. A major problem of the latter approach is that lesion boundaries are often overlapping in individual patients from different patient groups, thereby limiting the validity of such simple overlap group lesion studies (cf. [6]). Moreover, previous research on the behavioural effects of frontal brain damage often rested upon a comparison between groups of patients with lesions from many different etiologies (for a critical discussion see [10]).

To our knowledge, the VLBM method was applied for the first time to *FAB* performance in stroke patients.

## Method

### Subjects

Thirty-one acute first-ever, right-hemisphere-damaged stroke patients with frontal lobe involvement participated in the study (see Table 1 for details). The logic behind the restriction to right-hemisphere-damaged stroke patients was to exclude patients with a paresis of the dominant right hand and/or with apraxia, possibly distorting task performance of these patients due to impaired motor functions. Further, left-hemisphere strokes might have hampered the capability to understand task instructions, due to the potential presence of sensory aphasia.^a^ Patients with diffuse or bilateral brain lesions due to traumatic brain injury, brain tumors, subcortical arteriosclerotic encephalopathy, or any other dementing disease were excluded. Patients had no history of psychiatric disease or alcohol or drug abuse. Further, patients with gross neurological defects (pronounced pain as reported by the patient, left homonymous hemianopia as revealed by clinical examination, hemispatial visual neglect) were also excluded to make sure that these symptoms did not interfere with task performance.^a^ Spatial neglect was diagnosed when a patient showed the characteristic clinical behaviour such as orienting toward the ipsilesional side when addressed from the front or the left and/or ignoring contralesionally located people or objects. Table 1 shows demographic and neuropsychological participant characteristics.

**Table 1:** Demographic and neuropsychological patient characteristics

	***N***	***M***	***SD***
Age	31	59.61	10.31
Sex	31	19(m)/12(f)	/
Years of education	31	12.24	2.26
Handedness	31	0.93	0.26
CES-D [z]	23	0.06	0.86
MMSE [RS]	31	27.42	2.26
WST [z]	31	-0.36	0.83
RWT - subtest s-words [PR]	31	37.16	25.76
RWT – subtest animals [PR]	31	38.71	30.07
MCST - N categories [RS]	27	5.30	1.35
MCST - N perseveration errors [RS]	27	2.30	3.42

Center for Epidemiologic Studies Depression Scale, CES-D [11]; German version); handedness: handedness ratio on the Edingburgh Handedness Questionnaire ([12]; -1 = strongly left-handed, 0 = ambidextrous, 1 = strongly right-handed); Mini-Mental-State-Examination (MMSE [13]); Modified Card Sorting Test (MCST [14]); Regensburger Wortflüssigkeits-Test [Regensburger Word Fluency Test] (RWT [15]); Wortschatz-Test [Vocabulary Test] (WST [16]).

Note: Sex: m = male; f = female; years of education: school and vocational education; N = number of subjects; PR = percentile rank; M = Mean; RS = Raw Score; SD = Standard deviation; z = z-score.

### Standard protocol approvals, registrations, and patient consents

All patients gave their informed written consent to participate in the study, in accordance with the ethical standards of the Declaration of Helsinki (1964). Appropriate ethical approval for the study was obtained from the Ethics Committee at Technische Universität Braunschweig (Faculty for Life Sciences; Ref 37–2010).

### Test description, administration and scoring

The *FAB* consists of the following six tasks:

(1) **Similarities (conceptualization).** In this task, patients are required to identify the superordinate concept of two or more objects from the same semantic category. Specifically, patients were asked “In what way are the following objects alike?”: (1) a banana and an orange, (2) a table and a chair, and (3) a tulip, a rose, and a daisy. Only category responses (fruits, furniture, flowers) were considered correct. If patients achieved three correct responses, the score was 3; if they achieved two correct responses, the score was 2; if they achieved one correct response, the score was 1; if they achieved no correct response, the score was 0.

(2) **Lexical verbal fluency (mental flexibility).** This task requires the formation and exertion of self-organised cognitive strategies for efficient retrieval from semantic memory. It is well-documented in the neuropsychological literature that frontal lesions tend to decrease verbal fluency, particularly lexical verbal fluency [17,18], and that in right-handed people, unilateral right frontal lesions are related to the presence of noticeable deficits in lexical verbal fluency [17]. Patients were instructed to say in 60 seconds as many words as possible beginning with the letter *S*, any words that came to their mind except surnames or proper nouns. If patients achieved more than nine words, the score was 3; if they achieved six to nine words, the score was 2; if they achieved three to five words, the score was 1; if they achieved less than three words, the score was 0.

(3) **Motor series (programming).** This task requires the ability to program and execute a correctly ordered series of motor acts. Patients were asked to perform the Luria series ‘fist, edge, palm’ by initially copying the administrator three times, and then by repeating the series six times alone. If patients achieved six consecutive series by themselves, the score was 3; if they achieved at least three consecutive series on their own, the score was 2; if they failed at achieving at least three consecutive series alone, but achieved three when copying the examiner, the score was 1; otherwise the score was 0.

(4) **Conflicting instructions (sensitivity to interference).** This task challenges self-regulation in a behavioural interference paradigm by instructing patients to execute one action in response to the observation of a different action, thereby requiring the inhibition of imitative response tendencies [3,19,20]. Luria [2] had coined the term echopractic responses to signify his observation that patients with frontal lesions tend to display unintended imitative response tendencies. Patients were asked to hit the table once when the administrator hit it twice, or to hit the table twice when the administrator hit it only once. To ensure the patient had clearly understood the task, a practice trial was performed in which the examiner first hit the table once, three times in succession, and then twice, three more times. After the practice trial, the examiner completed the following series: 1–1–2–1–2–2–2–1–1–2. If patients made no errors, the score was 3; if they made one or two errors, the score was 2; for more than two errors, the score was 1, unless the patient copied the examiner at least four consecutive times, in which case the score was 0.

(5) **Go – Nogo (inhibitory control).** Patients were told that now, when the examiner hit the table once, they should also hit it once, but when the examiner hit twice, they should do nothing. To ensure the patient had clearly understood the task, a practice trial was performed in which the examiner hit the table once, three times in succession, and then twice, three more times. After the practice trial the examiner completed the following series: 1–1–2–1–2–2–2–1–1–2. If patients made no errors, the score was 3; for one or two errors the score was 2; for more than two errors the score was 1, unless the patient copied the examiner at least four consecutive times, in which case the score was 0.

(6) **Prehension behavior (environmental autonomy).** This task is designed to assess the tendency to activate patterns of behaviour that are involuntarily triggered by sensory stimulation, in some cases even against an explicit instruction not to show these activities. Following Dubois et al. [1], a particular sign of deficient environmental autonomy can be observed when the sensory perception (visual and/or tactile) of the experimenter’s hand compels patients to take them (prehension behaviour). The patient’s hands were placed palm up on the knees of the patient. The examiner touched both palms without saying anything. If the patient took the examiner’s hands, the examiner tried again after having asked the patient, not to take his hands. If patients did not take the examiner’s hands, the score was 3; if the patient hesitated and asked what to do, the score was 2; if the patient took the hands without hesitation, the score was 1; if the patient took the hands even after having been told not to do so, the score was 0.

The *FAB* global composite score was computed (range: 0 … 18) by summing up the six individual *FAB* task scores.

### Lesion analysis

Magnetic resonance imaging (MRI) was performed in 28 stroke patients and computed tomography (spiral CT) scanning was performed in three patients. The initial scanning was optionally repeated during the following days until the infarcted area became clearly demarcated. The mean time interval between lesion onset and the MRI scan that was used for the present analysis was 4.3 days (*SD* = 3.1); the mean time interval between time of lesion and CT scanning lasted 2.6 days (*SD* = 3.7). MRI scans were obtained on a 1.5 T echo planar imaging (EPI) capable system (Philips Intera, Philips Medical Systems, Best, The Netherlands). The MRI protocol used diffusion-weighted imaging (DWI, N = 12) and T2-weighted fluid-attenuated inversion-recovery imaging (FLAIR, N = 16). DWI was performed with a single-shot EPI spin echo sequence (25 axial slices; repetition times (TR), either 3690, 4000, 4452, 5060, 5300, or 6360 ms; echo times (TE), either 90, 95, or 120 ms; field of view (FOV), 230 × 230 mm^2^; matrix 64 × 64 pixels; slice thickness, 5 mm; gap, 5.5 mm). The FLAIR sequences were acquired with 25 axial slices (thickness, 5 mm) with an interslice gap of 5.5 mm, a FOV of 220 × 220 mm^2^, TR of either 4000, 5397, 5500, or 6000 ms, and TE of either 89, 91, 100, or 120 ms. CTs were obtained on a spiral scanning system (Somatom Sensation 16, Siemens Healthcare, Erlangen, Germany) with a slice thickness of 3 mm infratentorial and 6 mm supratentorial and an in-plane resolution of 0.5 × 0.5 mm.

Lesion location was evaluated using *MRIcroN* software ([7], http://www.mricro.com). For patients with MRI scans, the boundaries of lesions were delineated directly on the individual MRI scans. Both the MRI scan and the lesion shape were then mapped into stereotaxic space using the normalization algorithm provided by SPM5 (http://www.fil.ion.ucl.ac.uk/spm/software/spm5/). Cost–function masking was employed [21] for determination of the transformation parameters.

In patients with spiral CT scans, lesions were drawn directly by an experienced neurologist (H.-O. K.; blinded for test performance) on the slices of a normalized T_1_-weighted template MRI scan from the Montreal Neurological Institute (MNI) with a 1 × 1 mm in-plane resolution, distributed with the *MRIcroN* toolset. Lesions were mapped onto the slices that correspond to MNI Z-coordinates [-16, -8, 0, 8, 16, 24, 32, and 40 mm] by using the identical or the closest matching axial slices of each individual patient.

To evaluate the relationship between lesion location and performance on the *FAB*, a voxel-based lesion-behavior analysis was performed using the Liebermeister test implemented in the *MRIcroN* toolset [7]. The non-parametric Liebermeister test is performed on two binomial variables; it is a small-sample test for 2 by 2 tables. In the present context, one of the variables was ‘lesion present’ vs. ‘lesion absent’ in a particular voxel. Application of the Liebermeister test further requires patients to be assigned to two different groups based on a behavioural measure; given this, the Liebermeister test can identify voxels that when injured predict the presence of behavioral disturbance. The Liebermeister tests were based on median splits on the *FAB* global composite score and on the six individual *FAB* task scores (see Table 2 for the medians of the scores). Median splits were performed such that a “0” was assigned when task scores fell below the median (i.e., “0-2” for the items scores), whereas a score of “1” resulted from task scores that equalled or outranged the median (i.e., “3” for the item scores). Test statistics are maximum Liebermeister z-score (Lz) and critical Liebermeister z-score (z_crit_); Lz > z_crit_ indicates that there were voxels that when injured predicted the presence of behavioral disturbance.

**Table 2:** **Neuropsychological results and Liebermeister test statistics (maximum Liebermeister z-score, critical Liebermeister z-score) over various *FAB *** **scores**

***FAB score***	***M***	***SD***	***Mdn***	***IQR***	***max. Lz***	***z***_***crit***_
Global composite	15.06	3.00	16.00	4	3.435*	3.113
*FAB* 1	2.29	0.94	3.00	1	3.312*	2.966
*FAB* 2	2.48	0.89	3.00	1	3.784*	3.341
*FAB* 3	2.45	0.81	3.00	1	2.958	3.351
*FAB* 4	2.74	0.45	3.00	1	3.302	3.466
*FAB* 5	2.16	1.21	3.00	2	3.560*	3.143
*FAB* 6	2.94	0.36	3.00	0	2.278	2.278

Note: IQR = inter-quartile range (Q_75_-Q_25_); *p < .05.

Only voxels that were damaged in at least three patients were included in the analysis (*N* = 150.132 voxels). We controlled for multiple comparisons using permutation-based thresholding using 4000 iterations, as advocated in [7,22]. All results presented survived a 5% permutation-based false positive probability threshold.

## Results

### Neuropsychological test results on the FAB

Table 2 summarizes the performance of the patients on the *FAB*. The average *FAB* global composite score amounted to *M* = 15.06 (*SD* = 3.0). Task difficulty differed between the six *FAB* tasks, with *FAB* environmental autonomy being the easiest task and *FAB* inhibitory control being the most difficult task. The *FAB* conceptualizing score, the *FAB* mental flexibility score, and the *FAB* inhibitory control score showed relatively large variability compared to the *FAB* motor programming score, the *FAB* interference score, and the *FAB* environmental autonomy score.

Table 2 also summarizes the results obtained with the nonparametric Liebermeister test over all *FAB* scores *(FAB* global composite score and the six individual *FAB* task scores) to identify whether or not there were voxels that, when injured, were associated with the presence of behavioral disturbances on the *FAB*. Statistical significance was found for the *FAB* global composite score, the *FAB* conceptualizing score, the *FAB* mental flexibility score, and the *FAB* inhibitory control.

### Lesion analyses: lesion overlap

Figure 1 shows overlay lesion plots of all thirty-one patients in eight axial slices of a standard brain (i.e., in MNI space). Inspection of Figure 1 reveals that the maximum lesion overlap occurred in the right prefrontal cortex (PFC) where up to twelve patients showed overlapping lesions in single voxels.

**Figure 1:** **Overlay lesion plots of all thirty-one patients in *MNI *space.** Eight axial slices. The number of overlapping lesions is illustrated by colour, from violet (*N* = 1) to red (*N* = 31). Maximum overlap occurred in the right frontal lobe. The area coloured light blue indicates overlapping lesions in twelve patients (39% lesion overlap). Numbers indicate MNI coordinates.

### Lesion analyses: FAB global composite score

Figure 2 displays the results of a lesion subtraction analysis for global composite score. Figure 2A shows the overlay lesion plot of those patients who achieved a *FAB* global composite score below the median (*Mdn* = 16). The overlay lesion plot of those patients who achieved a *FAB* global composite score equal to or above the median is presented in Figure 2B. Figure 2C displays the results of a lesion subtraction analysis (patients below the median vs. patients equal to or above the median). The right frontal lobe was more frequently damaged in the group of patients who achieved low *FAB* global composite scores.

**Figure 2:** **Anatomical results obtained from the lesion subtraction analysis on the *FAB *global composite score. A**. Overlay lesion plots for those patients who achieved a *FAB* global composite score below the median (*Mdn* = 16; *N* = 15). The number of overlapping lesions is illustrated by colour, from violet (*N* = 1) to red (*N* = 15). **B**. Overlay lesion plots for those patients who achieved a *FAB* global composite score equal to or above the median (*Mdn* = 16; *N* = 16). The number of overlapping lesions is illustrated by colour, from violet (*N* = 1) to red (*N* = 16). **C**. Overlay plots of the subtracted superimposed lesions of the patients who achieved a *FAB* global composite score below the median minus patients who achieved a *FAB* global composite score equal to or above the median. Colours code increasing frequencies from dark red (difference 1% to 20%) to white-yellow (difference 81% to 100%), indicating regions damaged more frequently in patients who achieved a *FAB* global composite score below the median. The colours from dark blue (difference -1 to -20%) to light green (difference -81 to -100%) indicate regions damaged more frequently in patients who achieved a *FAB* global composite score equal to or above the median.

Figure 3A depicts the location of those voxels for which the voxel-based lesion-behavior analysis revealed a significant association between voxel damage and the *FAB* global composite score. This analysis revealed a small area around MNI coordinates X = 35, Y = 6, Z = 16, a sub-lobar gray matter coordinate within the anterior insula (BA13).

**Figure 3:** **Anatomical results obtained from the voxel-based lesion-behavior mapping (A) on the *FAB *global composite score, (B) on the *FAB *conceptualization score, (C) on the *FAB *mental flexibility score, and (D) on the *FAB *inhibitory control score.** The location of voxels for which the voxel-based lesion-behavior mapping indicated that the observed *Lz* surpassed *z*_*crit*_ is shown. See text for details. Numbers indicate MNI coordinates.

### Lesion analyses: FAB individual task scores

Figure 3B depicts the location of those voxels for which the voxel-based lesion-behavior analysis revealed a significant association between voxel damage and the *FAB* conceptualization score. Inspection of this map reveals that damage to lateral prefrontal subcortical brain areas is statistically associated with below-median performance in the *FAB* conceptualization score. Voxel-based statistical analysis revealed three regions: First, an area around MNI coordinates X = 32, Y = 6, Z = 16, a sub-lobar white matter coordinate near the anterior insula (BA13). Second, an area around MNI coordinates X = 28, Y = 15, Z = 24, a sub-gyral white matter coordinate near the claustrum. Third, an area around MNI coordinates X = 37, Y = 19, Z = 32, a sub-gyral white matter coordinate underneath the MFG (BA9).

Figure 3C depicts the location of those voxels for which the voxel-based lesion-behavior analysis revealed a significant association between voxel damage and the *FAB* mental flexibility score. Inspection of this map reveals that damage to lateral prefrontal subcortical brain areas is statistically associated with below-median performance in the *FAB* mental flexibility score. Voxel-based statistical analysis revealed an area around MNI coordinates X = 40, Y = 20, Z = 32, a white matter coordinate within the right MFG (BA9).

Figure 3D depicts the location of those voxels for which the voxel-based lesion-behavior analysis revealed a significant association between voxel damage and the *FAB* inhibitory control score. Inspection of this map reveals that damage to lateral prefrontal cortical and subcortical brain areas is statistically associated with below-median performance in *FAB* inhibitory control score. Voxel-based statistical analysis revealed two regions: First, an area around MNI coordinates X = 37, Y = 0, Z = 16 (also X = 31, Y = -2, Z = 24), sub-lobar white matter coordinates within near the anterior insula (BA13). Second, an area around MNI coordinates X = 53-58, Y = 7-18, Z = 8-16-24, sub-gyral white matter coordinates underneath the IFG (BA44/45).

The results from the remaining three FAB tasks (programming, sensitivity to interference, environmental autonomy) were negative.

## Discussion

Our voxel-based lesion-behavior mapping data give evidence to the proposition that *FAB* performance is sensitive to focal frontal lobe damage in the right cerebral hemisphere following stroke. Specifically, several *FAB* performance indices (i.e., *FAB* global composite score, *FAB* conceptualization score, *FAB* mental flexibility score, and *FAB* inhibitory control score) are significantly associated with the presence of lateral prefrontal lesions. Even more specifically, we found anatomical correlates of disturbed performance on the *FAB* global composite score, on the *FAB* conceptualization score, and on *FAB* inhibitory control score in or near the anterior insula (BA13). In addition to that, disturbed performance on the *FAB* mental flexibility score was related to lesions in the MFG (BA9), and performance on the *FAB* inhibitory control score was sensitive to damage of the right IFG (BA44/45). We did not, however, find evidence for a frontal contribution to performance on the *FAB* programming, on the *FAB* sensitivity to interference, and on the *FAB* environmental autonomy scores. Taken together, our voxel-based lesion-behavior mapping data support the proposition that some, yet not all, *FAB* measures are sensitive to lateral frontal lobe damage in the right cerebral hemisphere.

No earlier study was published which analyzed the effects of focal brain lesions following stroke on performance indices derived from the *FAB*, despite the fact that demonstrating the sensitivity of any neuropsychological measure to frontal damage is crucial to validating it as a suitable technique for assessing frontal functioning. Our voxel-based lesion-behavior mapping data fill this gap, providing initial evidence for the claim that performance indices on the *FAB* provide valid measures of frontal dysfunction.

The rapidly-growing literature on the *FAB* is mainly focused on two issues: First, on its capability to support the early diagnosis and differential diagnosis of neurodegenerative diseases (most notably the early diagnosis of bvFTLD as well as the differential diagnosis of bvFTLD and Alzheimer’s disease; [4,23-25]). In this realm, it is worth noting that degenerative brain atrophy affects most notably the anterior insular cortex during the earliest stages of the bvFTLD [26], suggesting that the sensitivity of *FAB* global performance for early-stage bvFTLD might be attributable, at least in part, to the anatomical association between *FAB* global composite score, *FAB* conceptualization score, *FAB* mental flexibility score, and *FAB* inhibitory control score and anterior insular dysfunction. Second, the capability of the *FAB* to detect executive dysfunctions in various diseases affecting fronto-striatal circuits constitutes a recent issue. Specifically, the *FAB* has been effectually used to document the presence of executive dysfunctions in various neurological diseases (e.g., amyotrophic lateral sclerosis [27,28]; Huntington’s disease [29]; multiple system atrophy and progressive supranuclear palsy [30]; Parkinson’s disease [31-34]) and psychiatric disorders (e.g., addictive substance abuse [35,36]; depression in Parkinson’s disease [37,38]). The results of the current study add to this rapidly-growing body of knowledge by strengthening the claim that various indices of *FAB* performance can be considered as valid assessments of lateral prefrontal, notably anterior insular, functioning.

There are three studies showing relationships between brain perfusion, as assessed by single photon emission computed tomography (SPECT), and *FAB* performance in patients suffering from various neurodegenerative diseases [39-41]. Although relationships between frontal perfusion and *FAB* performance have been consistently reported in each of these studies, the exact localization within the frontal lobes as well as the hemispheric lateralization of the anatomical basis of these relationships varied from study to study. A longitudinal study assessed MRI and behavioral measures of disease progression in FTLD [42]. Changes in *FAB* performance were associated with changes in whole brain MRI atrophy measures, though not uniformly across the three FTLD subgroups (i.e., bvFTLD, semantic dementia, progressive non-fluent aphasia).

Focal injuries to the right anterior insula (BA13) were associated with disturbed performance on the *FAB* global composite score, on the *FAB* conceptualization score, and on *FAB* inhibitory control score. These findings can hardly surprise, given the well-documented capability of the *FAB* to support the early diagnosis of bvFTLD (see above), and given the already mentioned relationship between degenerative brain atrophy in the anterior insular cortex during the earliest stages of the bvFTLD [24]. Further, anterior insula activations are often observed in functional neuroimaging studies, as detailed below.

The human anterior insular cortex participates in social-emotional processing (e.g., [43]). Other researchers have portrayed it as being part of a hedonic cortical network (e.g., [44]). According to Craig [45], ascending interoceptive pathways terminate in the posterior insula, whereas activation in the anterior insular cortex, possibly organized asymmetrically in an opponent fashion, correlates directly with subjective feelings from the body and with all emotional feelings. Lesions in the right posterior insula are associated with anosognosia for the functioning of one’s own limbs [46] and with the loss of the sense of limb ownership [47]. The right insular cortex seems to constitute a central node of a network involved in human body scheme representation [48].

The anterior insula/frontal operculum is also known to be involved in some basic cognitive functions. First, the right anterior insula/frontal operculum plays an important role in cognitive control [49-52], and the right anterior insula/frontal operculum seems to be involved in the control over the generation of appropriate behavioral responses to salient stimuli [53,54]. Second, activity in the anterior insula is related to the conscious perception of action errors, possibly enabling an orienting response when action errors are detected [55,56]. These relationships between activity in the (right) anterior insula and attentional control provide a possible explanation for the observed relationship between lesions in the right anterior insular cortex and *FAB* inhibitory control scores. Third, performance on tests of fluid intelligence produced extensive activity on the lateral frontal surface, in particular around the inferior frontal sulcus and anterior insula/frontal operculum in functional imaging studies (e.g., [57]), and lesions in these regions are associated with reduced fluid intelligence [58,59]. These relationships between activity in the anterior insula/frontal operculum and fluid intelligence provide a possible explanation for the observed relationship between lesions in the right anterior insular cortex and *FAB* conceptualization scores.

At first glance it may seem surprising that performance on *FAB* mental flexibility, actually reflecting lexical verbal fluency, was disturbed in stroke patients with injuries in the right frontal lobe. Henry and Crawford [17] reported strong evidence that lexical verbal fluency is more sensitive to frontal than nonfrontal lesions and left as opposed to right cortical lesions. Overall, their results were thus consistent with Ramier and Hecaen’s [60] suggestion that lexical verbal fluency performance is mediated by a verbal factor located in the left hemisphere and an executive component that reflects the integrity of the frontal lobes. When viewed from this perspective, the sensitivity of *FAB* mental flexibility scores to right frontal lesions reflects the degree of integrity of the executive component of lexical verbal fluency. This interpretation is further corroborated by our recent finding that injuries in similar areas of the right frontal lobe (i.e., BA9) are associated with deficient performance accuracy on *Form B* of the *Trail Making Test *[61] which requires to continuously switch back and forth between cognitive sets ([62]).

Further, it has extensively been documented in the literature on imaging and patient studies that the right IFG is closely related to response inhibition (e.g., [63-73]). Our finding contributes to this body of knowledge by showing that performance on the *FAB* Go – Nogo task, which is a simple clinical assessment technique for the ability to inhibit context-inappropriate responses, is actually sensitive to right IFG lesions in acute stroke patients.

## Conclusions

Our results show that specific aspects of *FAB* performance can be predicted from the presence of lateral prefrontal lesions, as discussed above. One could express the objection that a biased selection of patients entered the current study. Specifically, most study patients showed prefrontal lesions, whereas only a small number of patients with posterior lesions could be included in our study, thereby biasing the chance to detect reliable brain-behavior relationships in favour of prefrontal regions and to the disadvantage of posterior regions. It is important that we do not wish to claim that the hereby documented sensitivity of performance on the *FAB* towards prefrontal lesions is *specific* with regard to this particular lesion location. To date, solid information about the specificity of relationships between performance on the *FAB* and prefrontal lesions is not available. Another limitation of the current study is the lack of patients with lesions in the left hemisphere, thereby precluding any conclusion on hemispheric asymmetry. As noted by one of the reviewers, poor FAB composite or item scores could localize to areas within the left frontal lobe, but the present data cannot address this possibility.

Our findings are mainly reported in the white matter, while our discussion is essentially addressed on a cortical point of view and in relationship with previous findings in other pathological models. The FAB has formerly been validated on samples of patients with various neurodegenerative syndromes that affect several cortical and subcortical brain structures and white matter tracts. Although there was probably degeneration of frontal cortex in many of these cases, the pathology was clearly not restricted to the frontal cortex, raising the question whether the cognitive impairments observed could be ascribed solely or even primarily to frontal cortex damage. The difficulties in performance on the FAB might have been due to lesions in parts of the brain other than the frontal cortex, including multiple white matter regions. Here, we found disturbed performance on several FAB scores of patients who had damage limited to the frontal cortex and to no more than the immediately subjacent white matter. As it stands now, lesions of white matter subjacent to frontal cortex might be primarily responsible for the observed difficulties in performance on the FAB.

## Endnote

^a^A possible statistical solution to the problem would be to use the severity of hemiparesis, apraxia, aphasia, pain, hemianopia, neglect and other neuropsychological disturbances as covariates. However, covariance analysis presupposes the separation of patients into meaningful groups of individuals, as in neuropsychological group studies, and it further requires a number of restrictive conditions to be met such as, for example, that the slopes of the regression lines (which relate covariates and dependent variables), fitted to the groups, to be parallel.

## Abbreviations

BA: Brodmann’s area; bvFTLD: Behavioural variant of frontotemporal lobar degeneration; CES-D: Center for epidemiologic studies depression scale; CT: Computed tomography; DWI: Diffusion-weighted imaging; EPI: Echo planar imaging; FAB: Frontal assessment battery; FLAIR: Fluid-attenuated inversion-recovery imaging; FOV: Field of view; FTLD: Frontotemporal lobar degeneration; IFG: Inferior frontal gyrus; MCST: Modified card sorting test; MFG: Middle frontal gyrus; MMSE: Mini-mental-state-examination; MNI: Montreal neurological institute; MRI: Magnetic resonance imaging; PFC: Prefrontal cortex; RWT: Regensburger Wortflüssigkeits-test [Regensburger word fluency test]; SPECT: Single photon emission computed tomography; TE: Repetition time; TR: Echo times; VLBM: Voxel-based lesion-behavior mapping; WST: Wortschatz-test [vocabulary test].

## Competing interests

The authors declare that they have no competing interests.

## Authors’ contributions

BK contributed to the work by obtaining funding, designing the study, analyzing and interpreting the data, and drafting the manuscript. NR contributed to the work by acquiring and analyzing the data, and drafting the manuscript. ST contributed to the work by acquiring and analyzing the data. HJS contributed to the work by obtaining funding and drafting the manuscript. BdH contributed to the work by analyzing and interpreting the data, and drafting the manuscript. H-OK contributed to the work by obtaining funding, analyzing and interpreting the data, and drafting the manuscript. KW contributed to the work by obtaining funding and drafting the manuscript. All authors read and approved the final manuscript.

## Pre-publication history

The pre-publication history for this paper can be accessed here:

http://www.biomedcentral.com/1471-2377/13/179/prepub
